# Ageing in *Pgc-1β^−/−^* mice modelling mitochondrial dysfunction induces differential expression of a range of genes regulating ventricular electrophysiology

**DOI:** 10.1042/BSR20190127

**Published:** 2019-04-17

**Authors:** Charlotte E. Edling, Ibrahim T. Fazmin, Karan R. Chadda, Shiraz Ahmad, Haseeb Valli, Andrew A. Grace, Christopher L.-H. Huang, Kamalan Jeevaratnam

**Affiliations:** 1 Faculty of Health and Medical Sciences, University of Surrey, Guildford GU2 7AL, United Kingdom; 2 Physiological Laboratory, University of Cambridge, Downing Street, Cambridge CB2 3EG, United Kingdom; 3 Department of Biochemistry, Hopkins Building, University of Cambridge, Cambridge CB2 1QW, United Kingdom; 4 School of Medicine, Perdana University-Royal College of Surgeons Ireland 43400, Serdang Selangor Darul Ehsan, Malaysia

**Keywords:** cardiac arrhythmia, gene expression and regulation, ion channels, metabolic syndromes, Peroxisome proliferator activated receptor-γ coactivator-1

## Abstract

Mice deficient in mitochondrial promoter peroxisome proliferator activated receptor-γ co-activator-1β (*Pgc-1β^−/−^*) is a valuable model for metabolic diseases and has been found to present with several pathologies including ventricular arrhythmia. In the present study, our aim was to shed light on the molecular mechanisms behind the observed arrhythmic substrate by studying how the expression of selected genes critical for cardiac function differs in wild-type (WT) compared with *Pgc-1β* knockout mice and young compared with aged mice. We found that a clear majority of genes are down-regulated in the *Pgc-1β^−/−^* ventricular tissue compared with the WT. Although most individual genes are not significantly differentially expressed, a pattern is apparent when the genes are grouped according to their functional properties. Genes encoding proteins relating to ATPase activity, potassium ion channels relating to repolarisation and resting membrane potential, and genes encoding proteins in the cAMP pathway are found to be significantly down-regulated in the *Pgc-1β* deficient mice. On the contrary, the pacemaker channel genes *Hcn3* and *Hcn4* are up-regulated in subsets of the *Pgc-1β* deficient tissue. Furthermore, we found that with age, especially in the *Pgc-1β^−/−^* genotype, most genes are up-regulated including genes relating to the resting membrane potential, calcium homeostasis, the cAMP pathway, and most of the tested adrenoceptors. In conclusion, we here demonstrate how a complex pattern of many modest changes at gene level may explain major functional differences of the action potential related to ageing and mitochondrial dysfunction.

## Introduction

Cardiac arrhythmias result when the normal sequence of electrical activation and recovery in the heart is disrupted. Of the many arrhythmic variants the ventricular arrhythmias, particularly ventricular tachycardia and ventricular fibrillation, constitute the primary cause of sudden cardiac death, a common cause of mortality and a significant public health burden especially in the ageing population [1,2]. Major risk factors for ventricular arrhythmia and sudden cardiac death include age [3] and metabolic disorders [4,5] such as obesity, diabetes and metabolic syndrome. Metabolic conditions themselves are associated with mitochondrial dysfunction which in turn is strongly linked to cardiac arrhythmias suggesting that impaired mitochondrial capacity constitute a further link between metabolic disorders and cardiac arrhythmias [6].

Pgc-1β is one of the co-activators of peroxisome proliferator activated receptor-γ (PPARγ) that plays a pivotal role in controlling genes that are responsible for the regulation of lipid and glucose metabolism [7]. PPARγ and Pgc-1β are highly expressed in white and brown adipose tissues and in other oxidative tissues including cardiac and skeletal muscles [8] where it is a key regulator of basal mitochondrial function maintenance [9]. Pgc-1’s pivotal involvement in the cellular energy balance means that modifications of these actors has been proven to serve as useful experimental models for the analysis of pathological changes associated with energetic deficiencies such as metabolic disorders [10].

To study the independent and combined effect of age and metabolic disorders on ventricular arrhythmic substrate, we have employed the PPARγ co-activator-1β (Pgc-1β) knockout mice model [11]. In our previous studies we have explored action potential (AP) and pro-arrhythmic characteristics in intact Langendorff-perfused hearts from both young and aged, wild-type (WT) and *Pgc-1β^−/−^*mice [12–14]. We found that unprovoked young and aged *Pgc-1β^−/−^* hearts subject to a pacing protocol showed increased incidences of alternans in both AP activation (upshoot velocity and latency), recovery duration and resting membrane potential (RMP) compared with WT hearts, and aged *Pgc-1β^−/−^*hearts displayed increased incidence of actual arrhythmia. In conclusion *Pgc-1β^−/−^* hearts show pro-arrhythmic instabilities attributable to altered AP conduction and activation [14] and *Pgc-1β^−/−^*ventricular preparations showed consistently smaller Na^+^ currants independent of age even though other factors such as Na^+^ channel inactivation and K^+^ current activation were unchanged [15]. Moreover, morphometric assessments of the cardiac tissue indicated significantly increased fibrotic tissue with age and *Pgc-1β^−/−^* genotype [15].

In the present study, our aim was to explore the transcriptional activities in the ventricular cardiac tissue relating to arrhythmic risks associated with ageing and mitochondrial energetic dysfunction. We have selected a set of genes known to regulate the physiological processes underlying excitable activity leading to arrhythmia [2] and other genes considered markers for fibrosis, inflammation and other pathological changes impacting on the action potential generation. The genes have been grouped according to their physiological relevance as presented below.

### Na^+^–K^+^ ATPase activity

Na^+^–K^+^ ATPase α_1_ and α_2_ catalytic and accessory β_1_ subunits (encoded by *Atp1a1, Atp1a2* and *Atp1b1*) are related to the energetically dependent Na^+^–K^+^ ATPase-mediated membrane transport required to generate ionic gradients upon which the excitable activity is dependent.

### Ion channels relating to the resting membrane potential

The resting potential is mediated by background K^+^ channels. In this survey we have included a number of subtypes of ATP/ADP sensitive channels since we expect that the *Pgc-1β^−/−^* genotype causes intracellular ATP deficiency and hence sensitivity of potassium conductance to ATP/ADP is highly relevant. Genes included are the ATP-sensitive inward rectifier K^+^ channel Kir2.2 (*Kcnj12*) which links resting potentials to intracellular nucleotide levels [16], the ATP-binding cassette (ABC) transporter subunits members 8 and 9 (*Abcc8* and *Abcc9*), inwardly rectifying pore-forming K^+^ channels Kir6.1, Kir6.2 and Kir3.1 (*Kcnj8, Kcnj11* and *Kcnj3*) and G protein-activated inward rectifier potassium channel 4, Kir3.4 (*Kcnj5*). In addition we have included a gene representing Cl^−^ channel conductance, Clcn3, encoding the chloride voltage-gated channel 3.

### Ion channels relating to the initiation of excitable activity

In respect of the *Pgc-1β*^*−/*−^ mice resting heart rate and their response to chronotropic activation with adrenergic challenge we have included the *Hcn1, Hcn3* and *Hcn4* isoforms of hyperpolarisation-activated cyclic nucleotide-gated channels mediating SAN pacemaker currents I_h_ and the α units of the voltage-dependent Na^+^ conductances, *Scn5a* and *Scn7a*, to survey the initiation of excitable activity.

### Ca^2+^ homoeostasis – surface

To explore potential alterations in transcription of genes concerning the surface Ca^2+^ homeostasis we have included membrane voltage-dependent L-type Ca^2+^ channels Cav1.2 and Cav1.3 (*Cacna1c* and *Cacna1d*), T-type, Cav3.1 (*Cacna1g*) and Cav3.2 (*Cacna1h*), and the accessory β2 (*Cacnb2*), α_2_/δ1 (*Cacna2d1*) and α_2_/δ_2_ subunits (*Cacna2d2*).

### Ca^2+^ homoeostasis – intracellular

As well as surface Ca^2+^ homeostasis our survey covers molecules related to Ca^+^ homoeostasis between intracellular compartments. In this grouping we have included *Atp2a2* that encodes one of the SERCA transporter proteins regulating the cytosolic Ca^2+^ reuptake into the sarcoplasmic reticulum (SR), the principal cardiac Na^+^–Ca^2+^ exchanger NCX (*Slc8a1*), the SR Ca^2+^ binding protein calsequestrin (*Casq2*) and the ryanodine receptor isoforms RyR2 (*Ryr2*) and RyR3 (*Ryr3*) responsible for the SR Ca^2+^ release.

### Ion channels relating to repolarisation

Outward K^+^ currents regulate the action potential recovery phase that restores the transmembrane voltage to the resting potential level. These currents are mediated in murine hearts primarily by the voltage-sensitive transient outward current I_to_ carried by Kv1.4 and Kv4.3 (voltage-gated K^+^ channel subfamily A member 4 and subfamily D member 3, encoded by *Kcna4* respectively *Kcnd3*) [2]. We also include Kv11.1, another voltage-gated K^+^ channel (subfamily H member 2), encoded by *Kcnh2*, mediating the rapid K^+^ current, IKr, in view of its clinical importance [17]. Moreover, assays to survey the expression of *Kcnn1* and *Kcnn2* encoding the Ca^2+^-activated K^+^ channels KCa2.1 and KCa2.2, are included in this group since they are thought to contribute to the action potential repolarisation phase particularly in atria however also in ventricular tissue [18]. Lastly, we assayed expression of *Kcnk3* encoding the acid-sensitive K^+^ channel subfamily K member 3 and the regulatory KCNE1 subunit, encoded by *Kcne11*, in view of its association with some human Long QT syndromes [17].

### Adrenergic and cholinergic receptors

The autonomous nervous system innervate the cardiac tissue and cause the action potential to be generated in the sinoatrial (SA) node and the impulse then travels into the ventricles via the atrioventricular node (AV node). To explore potential alterations in this system we have chosen both α and β adrenergic and muscarinic cholinergic receptors to represent a complete repertoire of sympathetic and parasympathetic cardiomyocyte receptors including the pivotal β_1_ and β_2_-adrenergic receptor subtypes (*Adrb1* and *Adrb2*). In addition the α_1A_, α_1B_ and α_1D_ adrenergic receptor subtypes (*Adra1a, Adra1b* and *Adra1d*), are included since they are believed to have protective roles against pathological remodelling in heart failure [19]. *Chrm2*, muscarinic acetylcholine receptor type 2 is assayed as the main acetylcholine responsive receptor balancing against the adrenergic receptors.

### The cAMP pathway

As a consequence of adrenergic stimulation the cAMP (cyclic adenosine monophosphate) pathway is activated leading to calcium influx followed by increase in muscle contractility, heart rate, electrical conduction velocity and relaxation rate. To capture potential alterations in this principal cell signalling pathway we have explored cardiac adenylyl cyclase, types 4 and 5 (*Adcy4* and *Adcy5*), of which type 5 accentuates cardiomyopathic changes on chronic catecholamine stimulation, cGMP-dependent and cAMP-specific 3′,5′-cyclic phosphodiesterases 2A and 4D (*Pde2a* and *Pde4d*), the protein kinase A catalytic α-subunit (*Prkaca*), genes encoding the cAMP-dependent protein kinase regulatory subunits type I-α, II-α and II-β (*Prkar1a, Prkar2a* and *Prkar2b*) [20] and finally, we assay the major cardiac, calcium/calmodulin-dependent protein kinase, type II-δ (*Camk2d*), which mediates numerous cellular responses to Ca^2+^ signals [21].

### Fibrotic markers

In our previous physiological studies we have reported increased fibrotic change with age in mice with the *Pgc-1β^−^/^−^* genotype [22] and cardiac fibrosis is generally associated with altered cardiac conduction, (slowing, block and re-entry) [23]. In this study we examine fibrotic markers including the cytokine transforming growth factor β1 (TGF-β1*; Tgfb1*) [24], the gap junction forming protein δ 3, also known as Connexin 30.2 in mouse, encoded by *Gjd3*, the collagen precursor *Col3a1* encoding the collagen type III α1 chain and *Col1a1* encoding the major component of type I collagen, the fibrillar collagen found in most connective tissues [25].

### Other tested genes

The final group of genes tested are thought to act as markers for a range of developmental, inflammatory and hypertrophic changes ultimately impacting the AP generation and propagation. The transcriptional repressor Tbx3, encoded by *Tbx3*, is known to affect particular components of the cardiac conduction system, [26]. *Myh6* encodes the major thick filament protein MHC-α which is associated with late-onset hypertrophic cardiomyopathy and sinus node disorder if carrying mutations [2]. The cardiac hormone ANP (atrial natriuretic peptide), encoded by *Nppa*, is a known biomarker for heart disease, specifically, deficiency causes hypertension and cardiac hypertrophy which is related to its function as a regulator of the sodium balance. However recent studies has provided evidence that ANP also has a role in regulating vascular remodelling and energy metabolism [27]. The non-specific ion channel TRPC1 (*Trpc1*) conducts both Ca^2+^ and Na^+^ and has been found to be an important regulator of cardiac hypertrophy [28]. Finally in this miscellaneous group we have included genes encoding Pgc-1β itself and the complementary Pgc-1α (*Ppargc1b* and *Ppargc1a*).

## Materials and methods

### Animals

Experiments were approved by the University of Cambridge ethics review board under a U.K. project license for studies of cardiac arrhythmia. All procedures complied with the U.K. Home Office regulations (Animals (Scientific Procedures) Act 1986). The experiments also conformed to the Guide for the Care and Use of Laboratory Animals, U.S. National Institutes of Health (NIH Publication Number 85-23, revised 1996). Mice were housed in an animal facility at 21°C with 12-h light/dark cycles. Animals were fed sterile chow (RM3 Maintenance Diet, SDS, Witham, Essex, U.K.) and had free access to water, bedding and environmental stimuli. Mice were killed by cervical dislocation. No recovery, anesthetic or surgical procedures were required. WT C57/B6 and *Pgc-1β^−/−^* (The Jackson Laboratory, Maine, U.S.A.) mice were bred for the experimental protocols. Mice were bred on a C57/B6 background to avoid possible strain-related confounds.

### Tissue samples

The mice were divided into four groups: young WT (*n*=3), young *Pgc-1β^−/−^* (*n*=3), aged WT (*n*=3) and aged *Pgc-1β^−/−^* (*n*=3). Young mice were between the ages of 12 and 16 weeks and aged mice greater than 52 weeks. After extraction, the heart was cut to separate the ventricular tissue from the rest of the heart and subsequently snap-frozen.

### Taqman array assay

RNA was extracted from fresh frozen tissues, stored in −80°C, with the Qiagen RNeasy mini Plus kit. Cardiac ventricular tissue were weighed and quickly minced on ice. A third of the tissue, approximately 30 mg, was used in the next step of the RNA isolation protocol. The tissue was homogenised in RLT buffer supplemented with β-mercaptoethanol with a Stuart handheld homogeniser until completely smooth. Genomic DNA was eliminated by centrifugation through a column supplied with the kit prior to extraction of the RNA according to the manufacturer’s protocol. RNA integrity was assessed by using an Agilent Bioanalyzer to obtain RNA integrity numbers (RIN) according to the manufacturer’s protocol. RNA samples with RINs above 8 were used for the study. The RNA was used to prepare cDNA with High Capacity cDNA Reverse Transcription Kit (Applied Biosystems) according to the manufacturer’s instructions.

The efficiency of the cDNA protocol was tested by preparing the cDNA from a serial dilution of the RNA and then these cDNA samples were run with a SYBRgreen qPCR protocol confirming equal efficiency over a range of RNA concentrations. cDNA was also confirmed negative for genomic DNA contamination.

#### Thermo Fisher custom Taqman array cards

Each custom-made card contained 64 pre-validated assays in triplicate with a reaction volume of 1 μl. The cards were run exactly according to instructions specific for the cards. Briefly, the cDNA (100 ng/well) was mixed with 2× Mastermix from Thermo Fisher, 100 μl was loaded in each well slot on the cards, the cards were then spun down and sealed and run on a Quant 7 cycler. The amplification conditions were: 50°C for 2 min and 95°C for 10 min for the initial DNA melting and inactivation of the reverse transcription reaction, followed by 40 cycles of 95°C for 15 s and 60°C for 60 s.

Analysis of the Taqman array card data was performed by using the Quant studio software and Microsoft Excel by calculating fold changes with the delta-delta-*C*_T_ method [29]. The threshold was set at 0.2 fluorescence units and the baseline range was set to automatic assignment. The mean of the Cq values for the genes *HPRT, Gapdh* and *ActinB* were used as references.

### Statistics

*P*-values were calculated with Student’s independent *t*tests and Analysis of variance (Anova, one-way and two-way) and Tukey’s Honest Significant Difference (HSD) test where appropriate. Prior to *t*tests and Anovas the homogeneity of variance for the sample groups were tested with Levene’s test and were found negative (equal variance) for all groups. Statistical analyses were performed in the R programming language and statistical significance was assumed at *P*<0.05. Since our data to a high degree are exploratory with an aim to discover genes with differential expression we have opted to present the unadjusted *P*-values rather than with correction for multiple testing. We do acknowledge the risk of false positives and confirm that adjusting the *P*-values results in no statistical significance.

## Results

In the present study our focus has been to explore the effects on gene expression of both *Pgc-1β* deficiency and age at the individual gene level and as functional groups. To be able to analyse a large number of genes we used Custom Taqman array cards that were pre-probed with 60 cardiac function relevant genes as detailed above. The samples were divided into four groups: WT Young (*n*=3), WT Old (*n*=3), *Pgc-1β*^−/−^ Young (*n*=3) and *Pgc-1β^−/−^* Old (*n*=3).

To get a detailed overview of the differential expression of all tested genes Figure 1 present the raw expression fold changes as a heatmap with accompanying Anova single group and main effect significance statistics. The heatmap visualises the mean fold-changes for each tested group (Young-WT, Young-*Pgc-1β^−/−^*, Old-WT and Old-*Pgc-1β^−/−^*) at the individual gene level. At the top of the heatmap are the genes with the largest average decrease (green) in expression compared with the level in WT-Young samples (yellow) and at the bottom are the genes with the highest average increase in expression (red). As evident from the heatmap the majority of the investigated genes are relatively unchanged with both age and Pgc-1β deficiency, fold changes range from 0.38 to 2.06 compared with the WT-Young group. Two-way Anova main effect analyses however show a handful of significantly differentially expressed genes. The *Pgc-1β^−/−^* genotype significantly decrease the expression level of the ATPase activity regulating genes *Atp1a1* and *Atp1b1*, the adrenoceptor *Adra1d*, the potassium channels *Kcnj8* and *Kcnk3*, and *Casq2* encoding the calcium-binding protein Calsequestrin. The age factor significantly affects the level of the fibrotic marker *Col3a1*, potassium channels *Kcnj5* and *Kcnj3*, the pacemaker *Hcn3*, and the adrenoceptor *Adra1b*. Interestingly, all, but the fibrotic marker, are found to be up-regulated with age (Figure 1).

**Figure 1:** Heatmap visualising the differential expression Fold changes were normalised to the mean of the expression in WT/Young samples (*n*=3 for each group). The heatmaps show yellow for no change compared with WT/Young samples, red for increase and green for decrease in fold gene expression. The mean and the standard error of the mean (S.E.M.) are indicated for each biological group and gene. The genes are ordered in the direction of main change from largest decrease to largest increase compared with the WT/Young samples. Two-way ANOVA were performed to evaluate significance in differential expression between Young and Old respectively WT and *Pgc-1β^−/−^*. One-way ANOVA was performed to evaluate significance between all biological groups. Significance level *P*<0.05 are yellow marked for clarity.

In addition, the heatmap can be employed to distinguish genes where the effects of age and genotype are not necessarily substantially different however follow the same direction in the sense that the effect of age and genotype are potentially additive. We found five genes (*Nppa, Col3a1, Kcnn2, Trpc1* and *Col1a1*) that were consistently down-regulated with age and *Pgc-1β*^−/−^ genotype and we found two genes (*Hcn4* and *Gjd3*) that were consistently up-regulated with these factors (Figure 1). To further identify and analyse dependent interactions between age and *Pgc-1β* deficiency we also analysed the ‘between subject effects’ of the Two-Way Anova for age and *Pgc-1β*^−/−^. Only one gene, *Hcn3*, was identified as showing a significant (*P*=0.023) dependent interaction for the two tested factors. In this case that translates to that the expression change relating to age is dependent on the genotype and *vice versa*. For the other genes we found no significant dependencies between age and genotype nonetheless excluding the discussed general additive effects.

One-way Anova comparing the four groups (Young-WT, Young- *Pgc-1β*^−/−^, Old-WT and Old-*Pgc-1β*^−/−^) indicate significantly differentiating expression in only three genes (*Atp1b1, Kcnj3* and *Hcn3*) with Tukey’s HSD post hoc tests only pinpointing the pacemaker gene *Hcn3* in Old-*Pgc-1β*^−/−^ as being significantly different from the other groups (Old-*Pgc-1β*^−/−^ vs Young- *Pgc-1β*^−/−^; *P*=0.026 and Old-*Pgc-1β*^−/−^ vs Old-WT; *P*=0.045) (Figure 1).

To visualise and analyse the separate effects of age and genotype volcano plots displaying the magnitude of change against the level of statistical significance were produced by plotting the unadjusted *P*-values from pairwise-independent Student’s *t* tests against the log2 transformed expression fold changes for the *Pgc-1β*^−/−^ in young respectively Old mice (Figure 2A) and for the Old in WT respectively *Pgc-1β*^−/−^ mice (Figure 2B).

**Figure 2:** Pairwise gene expression ratios stratified by P-values (**A**) *WT* vs *Pgc-1β^−/−^* Volcano plots to show overview of differentially expressed genes in Pgc-1β^−/−^ tissue on single gene level grouped by age. Expression fold changes for Young-Pgc-1β^−/−^ were compared with Young-WT and Old-Pgc-1β^−/−^ were compared with Old-WT. *P*-values were calculated with unpaired Student’s *t*test. Genes with expression fold changes with *P*-value <0.10 are labelled in the plot. *n*=3 for each group. **(B)** *Young* vs *Old* Volcano plots to show overview of differentially expressed genes on single gene level grouped by Pgc-1β presence. Expression fold changes for WT-Old were compared with WT-Young and Pgc-1β^−/−^-Old were compared with Pgc-1β^−/−^-Young. *P*-values were calculated with unpaired Student’s *t*test. Genes with expression fold changes with *P*-value <0.10 are labelled in the plot. *n*=3 for each group.

Overall, the volcano plots confirm the heatmap analysis that the expression differences among the groups are relatively small and limited to a handful of genes. Even so, comparing WT with *Pgc-1β^−/−^* genotype in Young and Old mice separately clearly display that the majority of studied genes are less expressed in the *Pgc-1β* deficient mouse model in both Young and Old mice (Figure 2A). In young mice 54 out of 59 genes (not including *Ppargc1b*) were less expressed with an average decrease of 22%. In old mice the difference was less clear with 43 out of 59 genes less expressed with an average decrease of 9%. On single gene level five genes in the aged mice (*Atp1b1, Scn7a, Casq2, Kcnk3* and *Adra1*b) and none in the young mice were found to have significantly reduced gene expression in the *Pgc-1β^−/−^* genotype compared with normal as indicated in Figure 2A. Three of these genes, *Atp1b1, Casq2* and *Kcnk3*, were the same as found to be statistically different when assessed with Anova main effect analysis as well (Figure 1). Interestingly, when separating according to age it is evident that the statistical difference is bearing on the Old mice group and not found in Young mice. We also observed that the gene expression of the sodium ion channel encoded by *Scn7a* and the α-1 adrenergic receptor (*Adra1b*) were both significantly decreased in the aged mice however not in the young mouse population (Figure 2A).

In Figure 2B the expression levels of young and old mice in WT respectively *Pgc-1β* deficient mice are displayed in the same format as Figure 2A. Looking at these volcano plots it is evident that comparing tissue from young mice with aged mice (Figure 2B) show a significant increase in expression in aged mice, especially in the *Pgc-1β* knockout mice, where 45 out of 59 genes were more expressed with an average increase of 34%. In the WT group the difference was smaller with 40 out of 60 genes more expressed in old compared with young mice with an average increase of 11%. Despite the broadly increased expression levels in aged mice only three genes (*Kcnj3, Kcnj5* and *Hcn3*) in the *Pgc-1β^−/−^* mice, and none in the WT mice, were found to be significantly increased. As discussed above the *Kcnj3* and *Kcnj5* encodes potassium channel proteins important for the maintenance of the resting membrane potential and *Hcn3* is one of the hyperpolarisation-activated cyclic nucleotide-gated (HCN) channels that are vital for normal pace making.

In conclusion, the heatmap (Figure 1) and the volcano plots (Figure 2A) demonstrate that on a single gene level, there are a handful of genes that are significantly differentially expressed when comparing *Pgc-1β* deficient mice with WT in young and old mice. Even though most genes only show small changes in fold expression it is clear that knocking out *Pgc-1β* has a substantial effect on gene expression with an altogether significant decrease in expression of the studied set of genes. On the other hand, our data show that comparing the gene expression in young mice with old mice in both WT and mice with compromised mitochondrial function there is a general increase in gene expression with age in this particular set of genes (Figures 1 and 2B).

In the present study we have found that mitochondrial dysfunction and age both have relatively limited impact on the gene expression of our tested set of genes relevant for the cardiac action potential. At single gene level we have found a handful genes to be differentially expressed to a significance level *P*<0.05 as presented in Figures 1 and 2. To further explore the changes in gene expression pattern and potentially correlate these changes with the functional changes seen on the electrophysiological level [14,15,22] we have subgrouped the genes into ten groups according to their functions as indicated in Table 1 and discussed in the introduction.

**Table 1:** Functional group effects

		WT, Young mean	WT, Old mean	KO, Young mean	KO, Old mean	*Two-way Anova, significance*	
Genes	Functional groups	±S.E.M.	±S.E.M.	±S.E.M.	±S.E.M*.*	*Genotype*	Age
*Atp1a1, Atp1a2* and *Atp1b1*	Na^+^–K^+^ ATPase activity	1.00	1.01	0.58	0.72	*0.004*	*0.436*
		*0.06*	*0.10*	*0.05*	*0.12*		
*Kcnj12, Abcc8, Abcc9, Kcnj8, Kcnj11, Kcnj3, Kcnj5* and *Clcn3*	Ion channels relating to the resting membrane potential	1.00	1.19	0.82	1.06	*0.012*	*0.001*
		*0.03*	*0.06*	*0.05*	*0.08*		
*Hcn1, Hcn3, Hcn4, Scn5a* and *Scn7a*	Ion channels relating to the initiation of excitable activity	1.00	1.05	0.79	1.26	*0.994*	*0.153*
		*0.03*	*0.14*	*0.08*	*0.31*		
*Cacna1c, Cacna1d, Cacna1g, Cacna1h, cacnb2, Cacna2d1* and *Cacna2d2*	Ca^2+^ homoeostasis – surface	1.00	1.14	0.65	1.15	*0.173*	*0.014*
		*0.07*	*0.11*	*0.08*	*0.18*		
*Ryr2, Ryr3, Atp2a2, Slc8a1* and *Casq2*	Ca^2+^ homoeostasis – intracellular	1.00	1.27	0.85	1.08	*0.200*	*0.068*
		*0.05*	*0.13*	*0.07*	*0.21*		
*Kcna4, Kcnd3, Kcnh2, Kcnn1, Kcnn2, Kcnk3* and *Kcne11*	Ion channels relating to repolarisation	1.00	1.15	0.77	0.96	*0.018*	*0.055*
		*0.06*	*0.11*	*0.04*	*0.11*		
*Chrm2, Adra1a, Adra1b, Adra1d, Adrb1* and *Adrb2*	Adrenergic and cholinergic receptors	1.00	1.11	0.74	1.06	*0.102*	*0.027*
		*0.03*	*0.06*	*0.06*	*0.15*		
*Adcy4, Adcy5, Pde2a, Pde4d, Prkaca, Prkar1a, Prkar2b* and *Camk2d*	The cAMP pathway	1.00	1.05	0.85	0.94	*0.003*	*0.114*
		*0.03*	*0.04*	*0.05*	*0.05*		
*Tqfb1, Gjd3, Col1a2* and *Col3a1*	Fibrotic markers	1.00	0.99	0.86	0.96	*0.567*	*0.747*
		*0.11*	*0.14*	*0.08*	*0.21*		

Fold changes at gene level were first normalised to sample 1 of the WT-Young groups, then the means for the functional groups were calculated from the biological group means. The mean and the S.E.M. are indicated for each biological group of the functional groups. Two-way ANOVA were performed to evaluate significance in differential expression between Young and Old respectively WT and *Pgc-1β*^*−/*−^.

Two-way Anova main effect statistics for age and genotype show that four of the functional groups are significantly down-regulated comparing WT with *Pgc-1β*^−/−^ genotype and three of the groups are significantly up-regulated comparing Young with Old mice.

As a group the genes relating to the Na/K ATPase activity show a small but clear decrease in the *Pgc-1β* deficient group compared with WT in both young and old mice (Table 1). Also the ion channels relating to the resting membrane potential are, as a group, down-regulated in the *Pgc-1β*^*−/*−^ mice. On the contrary, comparing young with old mice there is a significant increase in gene expression of these genes again indicating changes of the resting potential maintenance however the genotypic changes are not additive to the effects of ageing. Exploring the genes relevant for the calcium homoeostasis we found only very minor changes. As presented in Figure 2A, the *Casq2* gene is slightly less expressed in old *Pgc-1β* knockout mice compared with WT. Genes regulating the calcium surface homoeostasis are not differentially expressed on the single gene level however as a group there is a significant increase with age. The same pattern was found when exploring the expression of the genes responsible for the repolarisation phase, at a single gene level only one gene showed a significant change in expression however as a group there is a statistical decrease in the *Pgc-1β^*−/*−^* genotype and also a distinct gene expression increase with age (Table 1). Adrenergic receptors mediating the sympathetic signalling in the cardiac tissue was found to be mainly down-regulated in our knockout model but then significantly increased as a group with age. The cholinergic receptor *Chrm2* showed the same pattern seemingly counteracting the adrenergic effects (the Anova group analysis is performed without the *Chrm2* gene expression). Following the gene expression changes of the adrenergic receptors the genes constituting the cAMP pathway are as a group significantly down-regulated with *Pgc-1β* deficiency and up-regulated with age even though at singular gene level the differences are considered non-significant. Lastly, studying our fibrotic markers as a group did not display any altered gene expression indicating that the decrease in the *Col3a1* with age discussed above might not be a general indicator of fibrotic change.

## Discussion

We have performed an extensive transcriptional profile of genes encoding molecules related to excitable activity (depolarisation, resting potential maintenance and repolarisation), calcium homoeostasis and fibrotic change which have been implicated in cardiac arrhythmias. Overall our aim has been to compare and relate the *Pgc-1β^*−/*−^* genotype and age-dependent phenotype with its transcriptional profile specifically regarding arrhythmic substrate, reductions in conduction velocity reflecting reduced Na^+^ current and increased tissue resistance.

The *Pgc-1β^*−/*−^* mouse model has proven to be a relevant model to study ‘metabolism induced’ arrhythmia [10,30]. Several previous studies [15,22,31,32] have explored the effects that this mitochondrial dysfunction has on the ventricular heart and it is now well established that mice deficient in *Pgc-1β* present with an age-dependent pro-arrhythmic phenotype. In the present study our aim was to investigate the molecular mechanisms causing this phenotype. We here describe how a set of genes known to determine the specifics of the AP and the cardiac conduction, including ion channels, fibrotic markers, cAMP pathway members and others, together form a complex pattern of regulation. We found that despite the clear physiological effects, the actual differences on gene level are relatively small. However, even though on single gene level the differential expression is minimal, we do find that grouping genes according to function shows a pattern of regulation. Interestingly, we found that, particularly in young mice, a vast majority of the studied genes are down-regulated in ventricular cardiac tissue from the *Pgc-1β^*−/*−^* mice. A natural explanation for this could be that since *Pgc-1β* deficiency causes the mitochondria to dysfunction and thereby lead to a lack of energy in the cell which in turn can cause lesser gene expression on the molecular level and arrhythmia on the functional level. Surprisingly though, with age, this same set of genes are mainly up-regulated, especially in the *Pgc-1β* deficient mice. It is possible that this up-regulation of gene expression is a compensation mechanism developed with age, however unlikely via *Pgc-1*α regulation since the level is unchanged across the samples.

We here suggest that the electrophysiological effects we have observed in the *Pgc-1β* deficient mouse model previously is potentially due to changes in gene expression of genes encoding proteins bearing on the Na–K ATPase activity (specifically *Atp1a1* and *Atp1b1*), the resting membrane potential (specifically *Kcnj3, 5* and *8*), repolarisation (specifically *Kcnk3*), the calcium balance (specifically *Casq2*) and proteins mediating the cyclic nucleotide signalling in response to autonomic activation. These groups of genes are to a high degree also involved in the changes seen with age pointing to that there might be overlapping mechanisms regarding ventricular arrhythmia in relation to metabolic disease and old age.

Characterisation of the action potential parameters by means of intact Langendorff-perfused hearts clearly point to increased pro-arrhythmic substrate in both older hearts and hearts with mitochondrial energetic deficiency [14,22]. For example the incidence of AP latency alternans was found to increase with age and *Pgc-1β^*−/*−^* genotype and the general frequency of actual arrhythmia was measured to be significantly higher in the aged *Pgc-1β^*−/*−^* hearts. However, even though initial ECG recordings showed shorter ventricular effective refractory periods (VERPs) for both young and aged *Pgc-1β*^*−/*−^ hearts with the aged *Pgc-1β^*−/*−^* heart markedly the shortest the following incremental pacing protocols indicated that the young, not old, *Pgc-1β^*−/*−^* hearts were least able to tolerate the shortened basic cycle length (BCL) at which hearts failed the pacing rate and entered block or ventricular arrhythmia. Moreover, both action potential duration (APD90) and the diastolic interval (DI90) was observed to be unchanged with age in the WT hearts however the APD90 was decreased in young *Pgc-1β^*−/*−^* hearts and increased in old *Pgc-1β*^−/*−*^ hearts and the DI90 was increased in the former and decreased in the latter compared with the level in the WT hearts [14,22]. Furthermore, regular 8 Hz pacing was conducted to resemble normal resting heart rate and action potential properties were characterised. Clear differences in maximum cardiac upstroke rate ((dV/dt)max) and AP duration were demonstrated. Interestingly both these factors were significantly dropped in Young *Pgc-1β*^−/−^ compared with young and old WT hearts however in the old *Pgc-1β*^−/−^ levels were picked up and even increased compared with WT hearts. The regular 8 Hz pacing did not cause spontaneous arrhythmic events in any of the experimental groups however with programmed electrical stimulation protocol a range of abnormal rhythms were elicited. Of particular interest was the counts of non-sustained ventricular tachycardia (NSVT) and sustained ventricular tachycardia (SVT). The latter was only recorded in the aged *Pgc-1β*^−/−^ however NSVT was significantly most frequent in the young *Pgc-1β*^−/−^ hearts [22].

Our aim with this transcriptional profiling study was to relate the physiological phenotypes of *Pgc-1β*^−/−^ and old age with the gene expression of targeted genes and our initial expectation was that mitochondrial dysfunction as a model for metabolic disease and ageing would be factors that independently and additively both increased the pro-arrhythmic substrate. Our data however indicate that the incidence of pro-arrhythmic substrate along with the gene expression follows a more complex pattern than anticipated. On a gene expression level the present data demonstrate that most genes are unchanged or changed only to a small degree and that age and mitochondrial dysfunction does not necessarily constitute additive effects. It is plausible that the effect of ageing and metabolic disorders, though similar, differs mechanistically on the molecular level. Interestingly, on a physiological level our previous data establish that ageing respectively metabolic disorder are not always mutually making symptoms worse indicating that there is indeed some congruence between gene expression and phenotype.

Considering the previously reported decrease in Na^+^ current and slowed conduction velocity we were surprised to find only the NaV2.1 (encoded by *Scn7a*) and not the main voltage-gated sodium channel NaV1.5 (*Scn5a*) to be down-regulated with age and mitochondrial dysfunction. Equally surprising we found no strong evidence that the previously described fibrotic activity was directly caused by transcriptional regulation. The two tested collagens in our study, *Col1a1* and *Col3a1*, are both marginally down-regulated, while the Gap Junction δ 2 protein, encoded by *Gjd3*, is up-regulated which at most suggest an imbalance in the fibrillar collagen regulation.

In conclusion we here provide evidence that the observed changes in the cardiac electrophysiology characteristics following ageing and mitochondrial dysfunction might be caused by a complex of surprisingly small transcriptional gene expression alterations. It is also possible that these observed changes are a consequence rather than a cause of the physiological changes and other yet unknown mechanisms control the pro-arrhythmic substrate.

## Abbreviations

Anova: analysis of variance
ANP: atrial natriuretic peptide
HSD: honest significant difference
Pgc-1β: promoter peroxisome proliferator activated receptor-γ co-activator-1β
PPARγ: peroxisome proliferator activated receptor-γ
RIN: RNA integrity number
SERCA: sarcoendoplasmic reticulum calcium transport ATPase
SR: sarcoplasmic reticulum
WT: wild-type

## References

[1] JosephsonM.E. (2014) Sudden cardiac arrest. Indian Heart J. 66, S2–S3 10.1016/j.ihj.2014.01.001 24568825PMC4237296

[2] HuangC.L. (2017) Murine electrophysiological models of cardiac arrhythmogenesis. Physiol. Rev. 97, 283–409 10.1152/physrev.00007.201627974512PMC5539373

[3] ChaddaK.R., AjijolaO.A., VaseghiM., ShivkumarK., HuangC.L. and JeevaratnamK. (2018) Ageing, the autonomic nervous system and arrhythmia: from brain to heart. Ageing Res. Rev. 48, 40–50 10.1016/j.arr.2018.09.005 30300712

[4] VasiliadisI., KolovouG., MavrogeniS., NairD.R. and MikhailidisD.P. (2014) Sudden cardiac death and diabetes mellitus. J. Diabetes Complications 28, 573–579 10.1016/j.jdiacomp.2014.02.003 24666923

[5] PlourdeB., SarrazinJ.-F., NaultI. and PoirierP. (2014) Sudden cardiac death and obesity. Expert Rev. Cardiovasc. Ther. 12, 1099–1110 10.1586/14779072.2014.952283 25160995

[6] YangK.-C., KyleJ.W., MakielskiJ.C. and DudleyS.C. (2015) Mechanisms of sudden cardiac death. Circ. Res. 116, 1937–1955 10.1161/CIRCRESAHA.116.304691 26044249PMC4458707

[7] JananiC. and Ranjitha KumariB.D. (2015) PPAR gamma gene - a review. Diabetes Meta. Syndr. Clin. Res. Rev. 9, 46–50 10.1016/j.dsx.2014.09.01525450819

[8] SonodaJ., MehlI.R., ChongL.-W., NofsingerR.R. and EvansR.M. (2007) PGC-1beta controls mitochondrial metabolism to modulate circadian activity, adaptive thermogenesis, and hepatic steatosis. Proc. Natl. Acad. Sci. U.S.A. 104, 5223–5228 10.1073/pnas.0611623104 17360356PMC1829290

[9] VillenaJ.A. (2015) New insights into PGC-1 coactivators: redefining their role in the regulation of mitochondrial function and beyond. FEBS J. 282, 647–672 10.1111/febs.1317525495651

[10] HandschinC. and SpiegelmanB.M. (2006) Peroxisome proliferator-activated receptor γ coactivator 1 coactivators, energy homeostasis, and metabolism. Endocr. Rev. 27, 728–735 10.1210/er.2006-0037 17018837

[11] LelliottC.J., Medina-GomezG., PetrovicN., KisA., FeldmannH.M., BjursellM. (2006) Ablation of PGC-1β results in defective mitochondrial activity, thermogenesis, hepatic function, and cardiac performance. PLoS Biol. 4, e369 10.1371/journal.pbio.004036917090215PMC1634886

[12] ChaddaK.R., AhmadS., ValliH., den UijlI., Al-HadithiA.B., SalvageS.C. (2017) The effects of ageing and adrenergic challenge on electrocardiographic phenotypes in a murine model of long QT syndrome type 3. Sci. Rep. 7, 11070 10.1038/s41598-017-11210-328894151PMC5593918

[13] ValliH., AhmadS., ChaddaK.R., Al-HadithiA.B.A.K., GraceA.A., JeevaratnamK. (2017) Age-dependent atrial arrhythmic phenotype secondary to mitochondrial dysfunction in Pgc-1β deficient murine hearts. Mech. Ageing Dev. 167, 30–45 10.1016/j.mad.2017.09.002 28919427PMC5652526

[14] AhmadS., ValliH., EdlingC.E., GraceA.A., JeevaratnamK. and HuangC.L. (2017) Effects of ageing on pro-arrhythmic ventricular phenotypes in incrementally paced murine Pgc-1beta-/- hearts. Pflugers Arch. 469, 1579–1590 10.1007/s00424-017-2054-328821956PMC5691113

[15] AhmadS., ValliH., SmythR., JiangA.Y., JeevaratnamK., MatthewsH.R. (2019) Reduced cardiomyocyte Na ^+^ current in the age-dependent murine *Pgc-1β ^−/−^* model of ventricular arrhythmia. J. Cell. Physiol. 234, 3921–3932 10.1002/jcp.2718330146680PMC6492124

[16] NicholsC.G. (2006) KATP channels as molecular sensors of cellular metabolism. Nature 440, 470–476 10.1038/nature04711 16554807

[17] SplawskiI., ShenJ., TimothyK.W., VincentG.M., LehmannM.H. and KeatingM.T. (1998) Genomic Structure of three long QT syndrome genes: KVLQT1, HERG, and KCNE1. Genomics 51, 86–97 10.1006/geno.1998.5361 9693036

[18] XuY., TutejaD., ZhangZ., XuD., ZhangY., RodriguezJ. (2003) Molecular identification and functional roles of a Ca(2+)-activated K+ channel in human and mouse hearts. J. Biol. Chem. 278, 49085–49094 10.1074/jbc.M307508200 13679367

[19] O’ConnellT.D., JensenB.C., BakerA.J. and SimpsonP.C. (2013) Cardiac alpha1-adrenergic receptors: novel aspects of expression, signaling mechanisms, physiologic function, and clinical importance. Pharmacol. Rev. 66, 308–333 10.1124/pr.112.007203 24368739PMC3880467

[20] TurnhamR.E. and ScottJ.D. (2016) Protein kinase A catalytic subunit isoform PRKACA: history, function and physiology. Gene 577, 101–108 10.1016/j.gene.2015.11.05226687711PMC4713328

[21] ZhangT., MiyamotoS. and BrownJ.H. (2004) Cardiomyocyte calcium and calcium/calmodulin-dependent protein kinase II: friends or foes? Recent Prog. Horm. Res. 59, 141–168 10.1210/rp.59.1.141 14749501

[22] AhmadS., ValliH., ChaddaK.R., CranleyJ., JeevaratnamK. and HuangC.L. (2018) Ventricular pro-arrhythmic phenotype, arrhythmic substrate, ageing and mitochondrial dysfunction in peroxisome proliferator activated receptor-γ coactivator-1β deficient (Pgc-1β−/−) murine hearts. Mech. Ageing Dev. 173, 92–103 10.1016/j.mad.2018.05.004 29763629PMC6004599

[23] SpachM.S. and BoineauJ.P. (1997) Microfibrosis produces electrical load variations due to loss of side-to-side cell connections: a major mechanism of structural heart disease arrhythmias. Pacing Clin. Electrophysiol. 20, 397–413 10.1111/j.1540-8159.1997.tb06199.x 9058844

[24] HaoX., ZhangY., ZhangX., NirmalanM., DaviesL., KonstantinouD. (2011) TGF-β1-mediated fibrosis and ion channel remodeling are key mechanisms in producing the sinus node dysfunction associated with SCN5A deficiency and aging. Circ. Arrhythm. Electrophysiol. 4, 397–406 10.1161/CIRCEP.110.960807 21493874

[25] DaviesL., JinJ., ShenW., TsuiH., ShiY., WangY. (2014) Mkk4 is a negative regulator of the transforming growth factor beta 1 signaling associated with atrial remodeling and arrhythmogenesis with age. J. Am. Heart Assoc. 3, 1–19 10.1161/JAHA.113.000340PMC418750824721794

[26] SylvaM., van den HoffM.J.B. and MoormanA.F.M. (2014) Development of the human heart. Am. J. Med. Genet. A 164A, 1347–1371 10.1002/ajmg.a.35896 23633400

[27] SongW., WangH. and WuQ. (2015) Atrial natriuretic peptide in cardiovascular biology and disease (NPPA). Gene 569, 1–6 10.1016/j.gene.2015.06.029 26074089PMC4496260

[28] OhbaT., WatanabeH., MurakamiM., TakahashiY., IinoK., KuromitsuS. (2007) Upregulation of TRPC1 in the development of cardiac hypertrophy. J. Mol. Cell Cardiol. 42, 498–507 10.1016/j.yjmcc.2006.10.020 17174323

[29] LivakK.J. and SchmittgenT.D. (2001) Analysis of relative gene expression data using real-time quantitative PCR and the 2−ΔΔCT method. Methods 25, 402–408 10.1006/meth.2001.1262 11846609

[30] RiehleC. and AbelE.D. (2012) PGC-1 proteins and heart failure. Trends Cardiovasc. Med. 22, 98–105 10.1016/j.tcm.2012.07.003 22939990PMC3466400

[31] AhmadS., ValliH., SalvageS.C., GraceA.A., JeevaratnamK. and HuangC.L. (2018) Age-dependent electrocardiographic changes in Pgc-1β deficient murine hearts. Clin. Exp. Pharmacol. Physiol. 45, 174–186 10.1111/1440-1681.1286328949414PMC5814877

[32] GurungI.S., Medina-GomezG., KisA., BakerM., VelagapudiV., NeogiS.G. (2011) Deletion of the metabolic transcriptional coactivator PGC1β induces cardiac arrhythmia. Cardiovasc. Res. 92, 29–38 10.1093/cvr/cvr155 21632884PMC3172981

